# Analysis of the Effect of the Integration Development of Sports Economy and Health Industry in the Context of Public Health Based on Big Data Analysis Technology

**DOI:** 10.1155/2022/1987918

**Published:** 2022-09-27

**Authors:** Liquan Chen

**Affiliations:** College of Sport Science and Physical Education, Mudanjiang Normal University, Mudanjiang, Heilongjiang 157012, China

## Abstract

In order to guide and meet people's health needs, various resources are flowing to the health sector, and the regional health economy is bound to develop rapidly, which increases the possibility of integrating and developing the sports economy and health industry in the context of the public health sector. As the health of the population improves, life expectancy increases, science and technology develops, and lifestyles change, the health economy sector is becoming increasingly active and both sport and healthcare will contribute to the development of the regional health economy. Big data, as a new management mindset and technical tool, brings new opportunities and challenges to the integrated development of sports economy and health industry. Based on the basic characteristics of big data, this paper provides a strategy for the development of the sports and health integration industry by using research methods such as grey correlation analysis, expert interviews, and agglomeration measures, starting from the problems faced by the integration development of China's sports industry to guarantee the construction of conditions. The experiment is analysed through the big data presentation of the health industry and the big data modelling ideas of grey correlation analysis, which provides new ideas to expand the application research of grey correlation analysis in the field of integration development.

## 1. Introduction

With the introduction of the Health China 2030 Plan, health economy has become a high-frequency term, and in 2011, the size of China's health economy exceeded 500 billion yuan [1]. The health economy is a collection of industrial activities such as production of products, provision of services, and dissemination of information on a large scale for the purpose of maintaining health, repairing health, and promoting health [2]. The health economy mainly aims to meet people's needs for health care to the maximum extent possible through the effective use of social resources and ultimately to promote and improve people's health. Therefore, health-related industrial activities are all related to the health economy. As an industry closely related to people's health, the sports industry has obvious health-related attributes. In recent years, the sports industry has gradually become a strategic emerging industry in China, playing an increasingly important role in the country's economic, scientific, and technological as well as humanistic development [3].

For the sports economy in public health to play a greater role in its implementation, it must integrate with other health industries and take the path of integrated development of the sports industry. But there are still many difficulties in how to better integrate with other industries and how to overcome them is the key. From a macro point of view, the prospect of integrating the sports industry and the health industry is indicated and planned as an important development path for the deep integration of national fitness and national health. At present, China's economy presents a new normal of transition from high-speed growth to high-quality development [4], and the population structure is moving from adult to elderly, with the Lewis inflection point [5]. In the context of the health concept and the construction of a strong sports nation, as a happiness industry that promotes people's well-being and enhances their growing aspirations for a better life, high quality has become the new connotation of the integration and development of the sports and health industries in the new era. How to improve the quality and efficiency of the integration of the two has important practical significance for improving the physical quality of China's nationals, adjusting the economic structure, and ensuring healthy economic development.

The sports industry is usually divided into four categories: sports goods manufacturing, professional sports, sports fitness, and leisure industry and related supporting services [6], which is a general term for a series of related economic activities centred on sports activities [7]. The sports industry is a collection of production activities that provide various sports products to the society with the ultimate goal of enhancing people's physical fitness and satisfaction and happiness in life, with the service industry as the main industry structure and the manufacturing industry as a supplement. There are two mainstream definitions of the health industry in the academic community. One is to divide the health industry into health manufacturing and health services according to the attributes of the products provided. The second is to divide the health industry into medical intervention health services and nonmedical intervention health services according to the mode and manner of service provision.

Industrial integration refers to the dynamic development process in which different industries or different sectors within the same industry interpenetrate and intersect with each other and eventually become one, gradually forming a new industry [8], including the comprehensive integration of technology, products, markets, talents, resources, and other aspects. Both the sports industry and the health industry have a wide range of people, comprehensive services, integration, and absolute positive externalities, and the industry involves a wide range of areas. Therefore, the high-quality integrated development of the sports industry and the health industry refers to a new model driven by new technologies, guided by meeting the people's growing need for a better life, based on the deep integration of national fitness and national health, and aiming at responding to the trend of people's consumption upgrade. Deep cross-fertilisation, interpenetration, and complementary advantages are carried out on the supply side of manufacturing and service industries to provide high-quality, high-efficiency, multilevel, and diversified products and services.

Since the 21st century, the progress of modern civilization has brought about an increase in the proportion of people with various chronic diseases and subhealth and an imbalance between health and income development, with rising living standards and declining health. While sport brings pleasure to people, it also promotes the development of a full cycle of health awareness, giving society a positive, stable, and orderly new look [9]. With the cross-border integration and interpenetration of industries as a new paradigm for high-quality economic development [10], the integration of sports and health industries will have more room for development and stronger market vitality. The national demand for health is growing at a high rate [11], and the content of sports and health consumption based on health care and recreation is in line with the people's goal of a green and healthy life. People are more willing to reduce their investment in mid-range disease treatment and gradually shift to the front-end national fitness and back-end rehabilitation and physiotherapy.

Technological advances and innovations often occur at the intersection of industries and change the products and market demand of the original industries, promoting deeper integration between industries. At this stage, as China's new infrastructure projects continue to be implemented, technologies such as 5G, big data, and the internet are moving into a new phase of development, bringing new opportunities for high-quality integration between the sports economy and the health industry, becoming the glue that holds the two together effectively. Promoting more specialisation and refinement of sports services and health services, new industries such as health data monitoring, smart venues, and intelligent health manufacturing have been derived, accelerating the interconnection of industry-wide ecology. At the same time, new technologies can further satisfy the public with diversified consumption demands, providing sports and health products of various types and rich content and forms. For example, in the field of exercise and health promotion, fitness centres can provide a variety of services that integrate sport and health for gym goers through new technologies. Related equipment manufacturers can also apply big data technology to smart wearable devices to form health interactions.

The rapid development of science and technology, such as the Internet, Internet of Things, cloud computing, and e-commerce, has given rise to huge amounts of semistructured and unstructured data in all areas of the economy and society, prompting huge challenges and new opportunities in the way of thinking and decision-making in modern management decision-making, while analysing and tapping the potential value of big data has become an important feature of modern management decision-making. On the other hand, as China's economy and society continue to progress and people's living standards continue to improve, the development of the big health industry has been brought to a strategic level by party committees and government departments at all levels. The new technologies introduced in the development of the industry have made the data of the big health industry gradually take on the characteristics of big data such as massive, multisource, heterogeneous, and low-density value.

Grey correlation analysis is an important element of grey system theory and has been widely cited by scholars in various research fields, such as the selection of regional strategic emerging industries [12], innovation efficiency analysis of high-tech industries [13], and the preferential selection of black-start schemes for power systems [14]. However, the application object of grey correlation analysis is the problem of information-poor uncertainty with little data, and its application area is “modelling of small sample data where some information is known and some information is unknown”. On the other hand, the era of big data has greatly increased the availability of all data or information in the field under study, which has also led to a crisis in the application of grey correlation analysis methods. The object of study of grey system theory should involve only poor information and not less data, i.e., the amount of data and poor information do not have a sufficiently necessary relationship, thus providing a theoretical basis for big data modelling of grey correlation analysis.

Some scholars initially explored the application research of grey correlation analysis in the era of big data, for example, Xu Lei studied the evaluation of efficient financial budget performance in the era of big data based on the improved model of grey correlation analysis [15]. Li et al. conducted a comprehensive assessment of electricity quality based on entropy power and grey correlation model and using electric power big data [16]. These two studies cover relevant aspects of big data but do not delve into big data modelling for grey correlation analysis, and they cover types of structured data without exploring modelling of semistructured and unstructured data. In view of the unique advantages and roles of grey correlation analysis methods in studying relevant factors of industrial development such as influencing factors, correlating factors, and controlling factors, exploring the integration development of sports economy and health industry is a positive contribution to the further development and improvement of grey system theory and so on. Based on the basic characteristics of big data and through the use of research methods such as grey correlation analysis, expert interviews, and agglomeration measurement, this paper proposes strategies for the development of the integrated sports and health industry from the perspective of the problems faced by the integrated development of China's sports industry, for the construction of guarantee conditions, the construction of incubation platforms, and the synergy between supply and demand.

## 2. Big Data Characteristics of the Sports Economy and Health Industry

The sports and health convergence industry is a general term for the industry that provides industrial, academic, and research products and related health services for the purpose of maintaining, improving, promoting, and managing health and preventing diseases [17]. Big data has 4 V characteristics, namely volume, variety, value, and velocity [18]. With the development of the Internet, the Internet of Things, cloud computing, and e-commerce, the data of the health industry has gradually acquired the four basic characteristics of big data. The path of high-quality integration and development of sports industry and health industry is shown in Figure 1.

### 2.1. The Massive Characteristics of Health Industry Data

The massive characteristics of health industry data are mainly manifested by the large amount of data and the rapid growth rate. With the rapid development of the Internet and the Internet of Things and the widespread use of barcode technology, data such as production and sales volume of big health products are constantly stored and used by manufacturers, intermediaries, logisticians, and sellers, prompting the rapid growth of data volume. Technologies such as telemedicine and wearable devices have enabled hospitals and health authorities to network the collection and use of data information such as patient signs, leading to a dramatic increase in data volumes. The characteristics of big data in the big health industry are (1) firstly, massive data can be obtained from the long time monitoring of the target objects; (2) massive data generated from the huge target groups; and (3) massive data derived from the many index attributes of the research objects.

The health management, medical rehabilitation, elderly care, and health and fitness industries are mainly for the general public, which inevitably involves a huge number of people. In 2016, China's elderly population aged 60 or above exceeded 230 million [19], and the number of people who choose elderly care institutions and smart home care is huge, thus generating a huge amount of data on elderly health. Currently, the number of people who are concerned about health and wellness is getting larger and younger, and the number of monthly active users of health and wellness through the Internet alone is over 10 million, which generates a huge amount of user data every day. In addition, the latest data from the State Food and Drug Administration shows that the number of health food products in China has reached 19,670.

The above facts indicate that the massive amount of data in the big health industry will be a primary feature of future activities such as industry management and decision-making. According to some sources, the health industry is expected to grow at an annual rate of 15% to 20% in the next 10 years, and the amount of data generated will grow exponentially.

### 2.2. Multiple Sources and Heterogeneous Characteristics of Health Industry Data

Big data comes from a wide range of sources, and its composition is diverse. The sources of data in the health industry include physiological, psychological, pathological, and therapeutic data collected by medical smart sensors and therapeutic devices; physical data on temperature, blood pressure, and heartbeat collected by smart wearable devices; data on temperature, humidity, wind direction, and pests from the health farming industry; and health products reflected in the media, markets, documents, and announcements.

The heterogeneity of data in the health industry is reflected in the media, marketing, documentation, and announcements. The heterogeneous nature of health data is reflected in the fact that information on health products in terms of form, quality, price, and geographical location can be stored in various forms such as text, images, videos, and websites. In addition to immediate information such as service price, service experience, body language, and quality satisfaction, the health service industry also has later information such as consumer credibility and audience reputation. It is clear that the diverse sources and heterogeneous storage methods of data in the health industry lead to great difficulties in processing the data.

### 2.3. The Low-Density Value Characteristics of Health Industry Data

There is no positive relationship between the value content of data and the total amount of data, which shows that only a small amount of data in the massive data can provide real value for managers' decision-making. As a result, it is more difficult for managers to obtain valuable information, and the amount of valuable information is diluted, so the massive data has obvious characteristics of low value density. The large amount of data obtained for infectious disease surveillance has little sensitive information and requires dynamic and continuous monitoring to capture abnormal information or discover its epidemiological pattern in such a huge amount of data. Inevitably, data bias and data errors occur during the management process of collection, storage, and replication. As a result, the large amount of daily information that the health industry obtains about its targets will inevitably lead to data bias and data redundancy, which will inevitably dilute the small amount of valuable information.

By forming a value chain with the main objective of jointly promoting the physical, mental, and emotional health and happiness of the masses as a link, promoting the integration of the cross and overlapping parts of the two industries, and extending and expanding the industrial space [20], the sports economy, which focuses on enhancing people's physical fitness and mental pleasure, and the health industry, which focuses on disease recovery and treatment, can be endogenously driven by the development of their respective advantageous industries. The development of in-depth integration within the industry to meet the diversified and differentiated health needs of consumers is shown in Figure 2.

## 3. Research Methodology

### 3.1. Grey Correlation Analysis

With the increasing penetration of big data into most industries in modern economic systems and most business functional areas in modern management activities, big data has become an important production factor and decision basis in modern production and management activities and has brought a crisis to the applied research of grey correlation analysis [21]. Big data modelling differs from traditional data modelling in its characteristics such as massive, multisource, heterogeneous, and low-density values, which bring significant challenges for grey correlation analysis models in terms of numerical adoption and computational accuracy.

In the study of grey correlation analysis, the main work is to establish grey correlation algorithm, and the algorithm model is mainly based on the following perspectives: reflecting the similarity of development process or magnitude between two series, reflecting the similarity of development trend or curve shape of two series, or considering the similarity and similarity of two series curves at the same time [22]. It is clear that the similarity or similarity features between the reference and comparison series of grey correlation coefficients and grey correlation modelling are easily cancelled out in the process of synthesis or merging when large amounts of data are used. In studying the process of model building between or within sequences, special attention should be paid to their differences from traditional data sequences.

In the healthcare industry, data can be broadly classified into four categories: data generated during patient visits, data from testing centres, data from pharmaceutical companies and gene sequencing, and data from smart wearable devices. Each type of data may differ in terms of the type or amount of data, and the sequence of data generated by each type of data may also differ to a certain extent. For the convenience of subsequent research, we establish a standard big data sequence form for the medical industry as follows.

(1) $$\begin{array}{c} Y_{i}=\left(t_{1},t_{2},\cdots ;p_{1},p_{2},\cdots ;v_{1},v_{2},\cdots ;a_{1},a_{2},\cdots ;\right)\left(i=1,2,3\cdots \right), \end{array}$$

where *t* is text data, *p* is image data, and *a* is audio data.

In this way, a number of large data series of the above types can form a system of medical health conditions for a patient. Based on the acquired data series, the management decision-maker can analyse the health status of the person and the factors influencing it.

In the process of studying big data sequences, the sequences differ from traditional data sequences in that they have a complex and diverse composition of elements, containing both numerical structured data and semistructured data such as web pages and unstructured data such as images, videos, audio, and location. As a result, big data sequences will cause a crisis in the application of grey correlation models.

In order to enable the big data sequences to be used effectively in constructing grey correlation analysis models, the big data sequences need to be. The data series should be preprocessed.

Assume that the big data sequences

(2) $$\begin{array}{c} X_{1}=\left(t_{1},t_{2},\cdots ;p_{1},p_{2},\cdots ;v_{1},v_{2},\cdots ;a_{1},a_{2},\cdots ;\right)\left(i=1,2,3\cdots \right). \end{array}$$

Dimensionless processing of data allows for the transformation of heterogeneous data into homogeneous data. After dimensionless processing large data series can be obtained as

(3) $$\begin{array}{c} X_{1}=\left(x_{1}^{t_{1}},x_{1}^{t_{2}},\cdots ;x_{2}^{p_{1}},x_{2}^{p_{2}},\cdots ;x_{3}^{v_{1}},x_{3}^{v_{2}},\cdots ;x_{4}^{a_{1}},x_{4}^{a_{2}},\cdots ;\right)\left(i=1,2,3\cdots \right). \end{array}$$

Through big data preprocessing, a grey correlation analysis model of big data can be attempted to be established. Referring to the traditional correlation model of grey correlation analysis theory, the grey correlation model between two data series in the big data environment can be constructed as follows.

(4) $$\begin{array}{c} \gamma \left(x_{1}\left(k\right),x_{2}\left(k\right)\right)=\frac{\text{minmin}\left|x_{1}\left(k\right)-x_{2}\left(k\right)\left|+\xi \text{maxmax}\right|x_{1}\left(k\right)-x_{2}\left(k\right)\right|}{\left|x_{1}\left(k\right)-x_{2}\left(k\right)\right|+\xi \text{minmin}\left|x_{1}\left(k\right)-x_{2}\left(k\right)\right|},\\ \gamma \left(X_{1},X_{2}\right)=\frac{1}{n}\overset{k}{\underset{n}{\sum }}\gamma \left(x_{1}\left(k\right),x_{2}\left(k\right)\right). \end{array}$$

Then, *γ*(*X*_1_, *X*_2_) is called the grey correlation between *X*_1_ and *X*_2_, where *k* is the *k*th element in the sequence and *ξ* is the discrimination factor.

To treat the elements of a large data sequence as a non-numerical sequence of the same structural type or to adjust only the positions of the data elements, then an appropriate multidimensional coordinate system can be considered to represent the data sequence, and then, a grey correlation model can be built with information on the possible positions of the coordinate system graphs, information on the possible composition of the angles, etc.

### 3.2. Expert Interview Method

Interviews and surveys will be conducted with experts, scholars, and relevant leaders in sports economy. A number of small symposiums will also be held to discuss the relevant issues of this paper and to consult with experts.

### 3.3. EG Index Measurement Method

Current methods of measuring industrial agglomeration include information entropy, industry concentration, locational Gini coefficient, spatial separation index, locational quotient, and kernel density estimation. In this paper, we adopt the EG index measurement method, and the specific steps are as follows:

**Step 1 .**

Calculation of locational Gini coefficient.

(5) $$\begin{array}{c} G_{i}=\overset{r=1}{\underset{R}{\sum }}{\left(X_{r}^{i}-X_{r}\right)}^{2}, \end{array}$$

where *R* is the number of cities, *X*_*r*_^*i*^ is the size of industry *i* in city *r* as a proportion of the size of that industry in all cities, and *X*_*r*_ is the size of all industries in city *r* as a proportion of the size of all industries in all cities. Clearly, indicator *G*_*i*_ reflects the degree of deviation of the geographical distribution of industry *i* relative to the geographical distribution of all industries. Under the condition of random distribution, the expected value of *G*_*i*_ is

(6) $$\begin{array}{c} E\left(G_{i}\right)=\left(1-\overset{\text{r}=1}{\underset{R}{\sum }}X_{R}^{2}\right)H_{\text{i}}. \end{array}$$

**Step 2 .**

Herfindahl index calculation.

Calculating the industry EG index requires first calculating the Herfindahl index *H* for that industry, and China does not keep statistics on the size of individual firms in an industry. Therefore, we use the estimation method of Yang Hongjiao [23], assuming that in each province, all enterprises within an industry have the same size, with the following estimation formula.

(7) $$\begin{array}{c} H_{i}=\overset{i=1}{\underset{P}{\sum }}\frac{{\left(X_{p}^{i}\right)}^{2}}{C_{p}^{\text{i}}}, \end{array}$$

where *P* denotes the category of province, *X*_*p*_^*i*^ is the size of industry *i* in province *P* as a proportion of the size of that industry in all provinces, and *C*_*p*_^i^ is the number of enterprises in industry *i* in province *P*. This method is the most accurate estimate given the availability of data.

**Step 3 .**

EG index calculation.

If firms choose their location randomly and the location choices are relatively independent, then the expected value of *γ* is zero. In this case, the advantages of nature, institutions, etc., have no influence on the location choice of enterprises. If the *γ* value of a neighbouring industry is greater than zero, the industry is spatially clustered and vice versa. The larger the *γ* value, the higher the concentration

(8) $$\begin{array}{c} \gamma_{\text{i}}=\frac{G_{\text{i}}-\left(1-\sum_{R}^{\text{r}=1}X_{r}^{2}\right)H_{i}}{\left(1-\sum_{R}^{r=1}X_{r}^{2}\right)\left(1-H_{\text{i}}\right)}. \end{array}$$

## 4. Analysis of Integration Development

### 4.1. Development of the Sports Economy

The current structure of China's sports economy is still unreasonable. In the USA, the flow of people, logistics, and services driven by professional sports competitions as the core has contributed to the economy of each state in the USA far more than one can imagine, and the impact of the sports economy on the economy of each state is very important and has now become one of the top ten industries in the USA [24]. As a result, state and local governments in the USA are spending considerable efforts to host sporting events and recruit related businesses [25]. Information on the total output and value added of China's sports economy in 2020 is given in Table 1.

A visual comparison of the total output and value added data for China's sports economy in 2020 is shown in Figure 3.

Figure 3 shows that the overall pattern of the sports economy in China has been formed, based on the manufacturing and sales of sports goods, driven by the sports competition and performance industry and the sports fitness and leisure industry, and the rapid development of sports venues, sports training, sports intermediation, and sports media. In the future, under the sustained effect of various policies, all relevant sectors of the sports economy will certainly usher in a period of rapid development. However, there are also problems such as the low total volume and the unreasonable internal structure of the sports economy, such as the high proportion of production and sales industries such as sports-related industries and the low proportion of sports services such as the sports industry.

In 2020, the total output of the sports economy in Beijing and Shanghai will be RMB 115.46 billion and RMB 104.59 billion, respectively, but the total output of three indicators representing the sports-based industry, namely sports competition and performance activities, sports fitness and leisure activities, and sports training and education, will be relatively low, as shown in Table 2.

A comparison of these sports economy figures for 2020 and 2021 is shown in Figure 4.

Figure 4 shows that the degree of agglomeration in the development of the sports economy is not yet high. Guided by the concept of fitness for all to health for all, the demand for health products will continue to increase for everyone as they grow older. In order to maximise the health needs of society at large, both developed and developing countries will continue to optimise the allocation of social resources, and health-related industries are bound to become areas where various resources are constantly concentrated, thus forming different degrees of agglomeration. A number of sports services and sports goods industry clusters have been formed in China, and industrial agglomeration has become a more important development model for the sports economy. In this situation, it has become inevitable to strengthen the management of the sports economy and realise the transformation of the sports economy development mechanism from management to governance, from control to performance, and from individual to synergy and the development of sports economy clustering.

The National Sports Administration has adjusted the caliber of sports economy statistics in 2021, but most provinces and municipalities have not yet done so. For the sake of consistency in the caliber of statistics and comparability of data, our collection of industry data started in 2018. For the purpose of analysis, based on the results of the expert interviews and the availability of data, the indicator of the number of employed persons in China's sports economy from 2018–2021 is selected for analysis in this paper. In this paper, industry employment wages are used to indicate the size of the industry, and the data source required for the calculation of the EG index is the number of employment wages by industry in each province and municipality, with a geographical scope of 31 provinces, municipalities, and autonomous regions. The number of fixed asset inputs by industry for the number of enterprises by industry in each province required to calculate the industry Herfindahl index is shown in Table 3.

The comparative effect of these five localities for the 2018–2021 sports economy EG index is shown in Figure 5.

Five provinces with a low EG industry index were also selected, and their specific data information is shown in Table 4.

A comparison of the data for these five provinces with low EG industry indices are shown in Figure 6.

From the calculation results in the table, it can be seen that, firstly, the degree of agglomeration of the sports economy in all Chinese provinces and cities is at a low level, with EG values generally less than 0.02. Secondly, from the perspective of each province and city, the degree of agglomeration of the sports economy is higher in Beijing and Shanghai, while the figures for other provinces are generally lower. Third, from the data of each province, the agglomeration development of the sports economy in each province of China shows a decreasing trend from 2018 to 2021. From the data calculated in this study, the sports economy has the highest degree of agglomeration, which also indicates that the development of China's sports economy has not been satisfactory compared to other industries in the past few years, and its concentrated development is obviously lagging behind that of other industries.

### 4.2. Development of the Health Industry

The current new medical model is able to cover a wide range of aspects and stages of healthy life. The characteristics of economic development have made the traditional mechanistic and biomedical models unable to adapt to the state of human health and are not meeting the quest for healthy conditions. This model is based on genetic, lifestyle, social, environmental, and psychological interventions, combining environmental, biological, psychological, social, and rehabilitation knowledge. With the emergence of this new medical model, more related industries will converge in the direction of health and the range of services will continue to expand. The sports economy, led by the concept of health, will not only expand in scale but will also become more prominent in its integration with the new medical model, with many industries converging and a huge industrial cluster about to be formed.

The position and role of the sports economy in the development of China's national economy has been increasing in recent years. The development of the sports economy has contributed to a new understanding of the goals, functions, and commercial attributes of sport in the academic world and has given rise to many new forms of sport and related industries, such as the health sports economy. The health industry EG index 2018–2021 is given in Table 5 for each province in China.

A comparison of the health industry EG indices for the five provinces in China for 2018–2021 is shown in Figure 7(a). The lower health industry EG index data for the five Chinese provinces for 2018–2021 is given in Table 6.

A comparison of the lower health industry EG indices for the five Chinese provinces from 2018 to 2021 is shown in Figure 7(b).

### 4.3. Integration of the Sports Economy and the Health Industry

The health industry and the sports economy both show the characteristics of convergence of value chains and cross-fertilisation of industries in the industrial chain, for example, sports and fitness services are an important part of the sports economy as well as an important service product of the health industry. Therefore, the sports economy and the health industry, with the ultimate goal of promoting the physical and mental health and pleasure of people, have a strong combination in the areas of disease and injury prevention and rehabilitation from the point of view of the continuity of the industrial chain and have formed a connection point between the two industrial value chains, the structure of which is shown in Figure 8.

At this linking point, there is a greater possibility for the sports economy to integrate with the health industry to develop new products, such as the integration of sport and health care, sport and physical function rehabilitation, sport and healthy ageing, sport and health advice, sport and nutrition, sport and health education, and many other aspects.

In summary, in terms of space, the products offered by the health industry cover a larger area than the sports economy, while in terms of time, the products offered by the sports economy are more advanced; compared to health issues, the products offered by the sports economy are more preventive; the sports economy highlights the function of enhancing human physical quality and mental pleasure at the front end of the value chain, while the health industry shows the function of treatment and rehabilitation at the back end of the value chain. The two are fused at the point of connection to form a sports-medicine fusion industry, which is more complementary in terms of health services.

The development of the sports-health integration industry should not only strengthen the synergy of all related industries within the sports economy but also achieve cross-industry synergy between industries, which requires that the theory of industrial synergy should be fully applied to promote the integration of China's sports economy and health industry. The key point is that the integration industry should take health and longevity as the ultimate goal, with the main functions including health maintenance for healthy people, health recovery for subhealthy people, and health repair for sick people, to create an industry chain covering the whole population and the whole life cycle, and the focus should be on the provision of integrated health services in the industrial scope.

Therefore, the guarantee system for the synergistic clustering of the physical and medical integration industry should be more complex than that of a single industry and should be a synergistic guarantee of good cooperation between the various guarantee systems. The construction of conditions for integration development needs to meet the following four points: (1) optimise top-level design and realise collaborative governance of government departments, (2) establish and improve relevant regulations and improve supervision and management mechanisms, (3) implement inclined monetary and financial policies and use credit leverage to support the development of the integrative health industry, and (4) develop human capital for the development of the integrative health industry.

## 5. Conclusion

With the improvement of national health level and the extension of life expectancy per capita, the development of science and technology, and the change of lifestyle, the field of health economy is increasingly active, and both sports and medical care will play a role in promoting the development of regional health economy. The development of the sports and medical integration industry is still at the beginning stage, and the characteristics of agglomeration development are not yet obvious. This paper explores the big data modelling problem of grey correlation analysis using health industry data as an example, giving preprocessing methods and grey correlation modelling ideas for big data modelling. It also uses expert interviews and agglomeration measures to conduct research to achieve the collaborative agglomeration development of the health care integration industry in terms of guaranteeing the construction of conditions and analyses the specific strategies for integration development. The method proposed in this paper is a summary and sublimation of the theory of industrial agglomeration and cluster evolution, which is of great significance as a guide to the convergence development of related industries in China.

## Figures and Tables

**Figure 1:** The path to high-quality integration of the sports economy and the health industry.

**Figure 2:** Space for the integration of sports economy and health industry sectors.

**Figure 3:** Comparison of data on total output and value added in China's sports economy in 2020: (a) total output and (b) value added.

**Figure 4:** Sports economy data for 2020 compared to 2021.

**Figure 5:** Comparison of the EG index for the sports economy, 2018–2021.

**Figure 6:** Comparison of data from the five provinces with lower EG index for sports economy, 2018–2021.

**Figure 7:** Comparison of lower health industry EG indices in five Chinese provinces: (a) higher index and (b) lower index.

**Figure 8:** Structure of the integration of the sports economy and the health industry.

**Table 1:** Total output and value added of the sports economy in China in 2020.

Sports industry category	Total output	Value added
Sports management	287.1	143.8
Sports competition	176.8	65.5
Physical fitness	368.6	175.6
Gym	523.5	256.3
Sports intermediary	156.3	114.2
Sports training	296.8	230.5
Sports media	145.2	144.3
Sports-related services	532.2	178.5
Sporting goods	852.3	368.3
Sports facilities	263.5	127.8

**Table 2:** Survey of sports economy income in Beijing and Shanghai, 2020–2021.

Projects	2020		2021	
	Beijing	Shanghai	Beijing	Shanghai
Sports management	32.3	31.4	27.8	26.3
Sports competition	89.2	35.7	70.6	23.4
Physical fitness	33.9	45.7	34.7	40.4
Gym	37.1	18.2	28.9	15.6
Sports intermediary	36.3	15.2	26.3	16.8
Sports training	17.6	17.3	19.8	12.5
Sports media	69.9	60.5	62.5	31.1
Sports-related services	85.3	59.9	75.6	41.8
Sporting goods	68.4	70.5	65.9	56.4
Sports facilities	26.8	35.7	19.8	15.5

**Table 3:** 2018–2021 EG index for the sports economy in the five regions.

Province	2018	2019	2020	2021
Beijing	0.018	0.016	0.015	0.013
Shanghai	0.015	0.014	0.013	0.014
Hebei	0.003	0.004	0.003	0.004
Tianjin	0.002	0.003	0.002	0.002
Shanxi	0.002	0.001	0.001	0.002

**Table 4:** Data for the five provinces with a lower EG index for the sports economy, 2018–2021.

Province	2018	2019	2020	2021
Gansu	0.00027	0.00025	0.00023	0.00021
Qinghai	0.00018	0.00016	0.00015	0.00013
Ningxia	0.00025	0.00024	0.00021	0.00019
Xinjiang	0.00035	0.00037	0.00036	0.00032
Xizang	0.00018	0.00015	0.00013	0.00014

**Table 5:** Health industry EG index by province in China, 2018–2021.

Province	2018	2019	2020	2021
Beijing	0.00045	0.00035	0.00032	0.00028
Shanghai	0.00021	0.00020	0.00018	0.00014
Hebei	0.00015	0.00013	0.00011	0.00010
Tianjin	0.00010	0.00011	0.00014	0.00016
Shanxi	0.00017	0.00015	0.00014	0.00012

**Table 6:** Lower health industry EG index for five provinces in China, 2018–2021.

Province	2018	2019	2020	2021
Gansu	0.00009	0.00008	0.00007	0.00005
Qinghai	0.00003	0.00002	0.00003	0.00001
Ningxia	0.00007	0.00005	0.00004	0.00003
Xinjiang	0.00002	0.00003	0.00005	0.00006
Xizang	0.00006	0.00005	0.00003	0.00002

## Data Availability

The dataset can be accessed upon request.
